RETRACTED

# Adaptive Anomaly Detection Framework Model Objects in Cyberspace

**DOI:** 10.1155/2020/6660489

**Published:** 2020-12-09

**Authors:** Hasan Alkahtani, Theyazn H. H. Aldhyani, Mohammed Al-Yaari

**Affiliations:** ^1^College of Computer Science and Information Technology, King Faisal University, P.O. Box 4000, Al-Ahsa 31982, Saudi Arabia; ^2^Community College of Abqaiq, King Faisal University, P.O. Box 4000, Al-Ahsa 31982, Saudi Arabia; ^3^Chemical Engineering Department, King Faisal University, P.O. Box 380, Al-Ahsa 31982, Saudi Arabia

## Abstract

Telecommunication has registered strong and rapid growth in the past decade. Accordingly, the monitoring of computers and networks is too complicated for network administrators. Hence, network security represents one of the biggest serious challenges that can be faced by network security communities. Taking into consideration the fact that e-banking, e-commerce, and business data will be shared on the computer network, these data may face a threat from intrusion. The purpose of this research is to propose a methodology that will lead to a high level and sustainable protection against cyberattacks. In particular, an adaptive anomaly detection framework model was developed using deep and machine learning algorithms to manage automatically-configured application-level firewalls. The standard network datasets were used to evaluate the proposed model which is designed for improving the cybersecurity system. The deep learning based on Long-Short Term Memory Recurrent Neural Network (LSTM-RNN) and machine learning algorithms namely Support Vector Machine (SVM), K-Nearest Neighbor (K-NN) algorithms were implemented to classify the Denial-of-Service attack (DoS) and Distributed Denial-of-Service (DDoS) attacks. The information gain method was applied to select the relevant features from the network dataset. These network features were significant to improve the classification algorithm. The system was used to classify DoS and DDoS attacks in four stand datasets namely KDD cup 199, NSL-KDD, ISCX, and ICI-ID2017. The empirical results indicate that the deep learning based on the LSTM-RNN algorithm has obtained the highest accuracy. The proposed system based on the LSTM-RNN algorithm produced the highest testing accuracy rate of 99.51% and 99.91% with respect to KDD Cup'99, NSL-KDD, ISCX, and ICI-Id2017 datasets, respectively. A comparative result analysis between the machine learning algorithms, namely SVM and KNN, and the deep learning algorithms based on the LSTM-RNN model is presented. Finally, it is concluded that the LSTM-RNN model is efficient and effective to improve the cybersecurity system for detecting anomaly-based cybersecurity.

RETRACTED

## 1. Introduction

The end of the Cold War has led to many challenges and threats that the international community has never seen before, known as asymmetric or asymmetric cross-border threats that recognize neither borders and national sovereignty nor the idea of a nation-state. These threats led to shifts in the field of security and strategic studies as well as at the level of political practice. The explosion of the information revolution and the entry of the digital age, especially in the 21st century resulted in many repercussions manifested in the emergence of cyber threats and crimes. Such threats are regarded to be a major challenge to the national as well as international security making cyberspace as the fifth area of war after land, sea, air, and space. These repercussions entailed the need for security guarantees within this digital environment which led to the emergence of cybersecurity as a new dimension within the field of security studies that has acquired the interests of many researchers in this area. Having said that, we need to understand what cybersecurity is as a new variable in international relations. The task of adjusting concepts and terminology is a challenge facing various researchers and scholars in different disciplines because of the problems it poses making it difficult to agree on clear, comprehensive, and unified definitions among members of the scientific community. Cybersecurity is one of the complex concepts that have been presented by many different definitions. In this sense, researchers in the field of international relations and other subfields in security and strategic studies are increasingly focusing on the impact of technology on national and international security, including related concepts such as power and sovereignty, global governance, and securitization. As a matter of fact, the expansion of the internet has reshaped traditional forms and norms of the international force that are working extensively to enter a new era of geopolitics.

Cybersecurity is the technical, regulatory, and administrative means that are used to prevent unauthorized use, abuse, and recovery of electronic information over communication systems and the information they contain. In addition, the aim of cybersecurity is to ensure the availability and continuity of the work of information systems and enhance the protection, confidentiality, and privacy of personal data by all measures. Cybersecurity is the practice of defending computers, servers, mobile devices, electronic systems, networks, and data from malicious attacks, also known as information security or cyberwarfare [1]. One of the major challenges of network traffic analysis is intrusion detection. The Intrusion Detection Systems (IDS) are designed to find out malicious activities that attempt to compromise the confidentiality, integrity, and assurance of computer systems. The intrusion detection system has become the most widely used security technology [2]. Certainly, intrusion detection systems have become critical components in network security. Consequently, two factors need to be considered to guarantee an effective performance of IDS. First, the intrusion detection should deliver consistent detection results. The detection method should be effective in discovering intrusions since poor detection performance ruins the trustworthiness of the IDS. Second, the IDS should be able to survive in hostile environments (i.e., under attacks). The main challenge for IDS is to maintain high detection accuracy. As new intrusions increase, IDS tools are becoming incapable of protecting computers and applications. Consequently, a robust approach that is able to discover new attacks is necessary for building reliable IDS. Machine learning provides insights for identifying novel attacks. Machine learning enhances the capability of a machine that automatically improves its performance through learning from experience [3–7]. Machine learning techniques are employed to study normal computer activities and identify anomalous behaviors that deviate from the normal as intrusions. Even though these anomalies-based IDSs are able to detect novel attacks, most of them suffer from misclassification.

RETRACTED

The algorithms of machine learning have played a crucial role in the area of cybersecurity. Deep learning networks performed incredibly in solving problems from a wide variety of fields. Furthermore, as can be observed, it gained a significant increase in its usage for artificial intelligence (AI) and unsupervised challenges [8]. The artificial neural network is part of machine-learning simulating the processes of the human brain. Deep learning refers to simple building blocks that are organized in a complex hierarchical order. These building blocks have the ability to solve high-level problems. Recently, the applications of deep learning methods are oriented towards various uses, especially cybersecurity [9–11]. In recent years, deep learning has evolved as an important research area in machine learning. Viewing it as a special architecture of deep learning, DNN has proved to be of effective applications, particularly in different tasks of pattern recognition such as visual classification and speech recognition. Having said that, recent studies from 2013 onwards have shown that DNN is prone to serious attacks [12, 13]. An example that shows the vulnerability of DNN is image classification where it extracts only few features which hinder its performance, especially with images that have nuanced differences. Thus, it is easy for attackers to evade anomaly detection. Szegedy et al. [12] suggested using a slightly blurred image to trick the pretrained DNN. This was followed by many works that suggested impersonation models for the sake of attacking DNNs and proposing corresponding intelligent systems (e.g., face recognition, speech recognition, and autonomous driving) [14–17]. Fiore et al. [18] explored the use of a semisupervised model for network intrusion detection. They used a discriminative restricted Boltzmann machine to combine the expressive power of generative models with good classification abilities. They employed the KDD Cup'99 dataset with a set of 41 features and 97,278 instances. Salama et al. [19] paired the Restricted Boltzmann Machine (RBM) with Support Vector Machine (SVM) to build a traffic intrusion detection system.

RETRACTED

The dataset used in the study was NSL-KDD, and its training set had a 22 training attack types along with 17 types in the testing set. The study demonstrated that such combination showed better performance in classification compared to the classification of support vector machine alone. Alrawashdeh and Purdy [20] implemented the RBM with a deep belief network for anomaly detection. They employed the KDD Cup'99 dataset which consisted of 494,021 training records and 311,029 testing records. They carried out the deep learning architecture in C++ in Microsoft Visual Studio 2013. Their study demonstrated that the use of a Restricted Boltzmann Machine improved the accuracy of classifying attacks to 92%. The article showed better results than those implemented by Salama et al. [19] in both accuracy and speed detection. Aldwairi et al. tested the effect of appropriate features on the performance of Restricted Boltzmann Machines and compared its performance with conventional machine learning algorithms [21]. Their study demonstrated that Restricted Boltzmann Machines can be trained to accurately classify and distinguish between normal and anomalous Net Flow traffic. The study employed the ISCX dataset [22] and applied it in the intrusion detection area. They employed a restricted Boltzmann machine in which its deep neural network training is made of two steps: (i) training restricted Boltzmann machine, and (ii) tuning the parameters of the whole RBM. The results demonstrated that using the restricted Boltzmann machine on the KDD Cup'99 dataset of deep belief network outperformed the performance of a support vector machine and an artificial neural network. Fu et al. [23] improved a framework for detecting fundamental patterns of deceptive behaviors, such as the detection of fake credit cards. The framework is based on the convolutional neural network. The convolutional neural network was also implemented by Zhang et al. [24]. They used the data of the commercial bank B2C online transactions. The transaction data of one month were classified into training and testing datasets. The results showed an accuracy rate of 91% and a recall rate of 94%. Compared with the results of Fu et al. [23], the results of Zhang et al. showed an increase in the accuracy and recall rate with 26% and 2%, respectively. Nasr et al. designed a particular system that is called DeepCorr which is based on deep learning architecture to learn a flow correlation function tailored to Tor's complex network. In their experiment, DeepCorr achieved the best performance with a learning rate of 0.0001, and for a false-positive rate of 10-3, achieved a true positive rate close to 0.8. Zhang et al. designed an anomaly traffic detection model leveraging two layers of the neural network [25]. The first layer is made of the improved LetNet-5 convolutional neural network with the function to extract the spatial features. The second layer makes use of long short-term memory with the function to extract temporal features. On the CIC-IDS2017 dataset, the performance exceeded 94%. Their suggested system achieves better accuracy, F1-measure, and higher recall rate compared to other machine learning algorithms. Thus, the framework proposed by Zheng et al. is regarded as light-weight with the ability to detect new attacks and classify encrypted traffic. Yu et al. applied a convolutional autoencoder to test the efficiency of the detection system on network intrusion [26]. Two datasets were employed: they are the CTU-UNB and Contagio-CTU-UNB. To develop the neural network model, the Theano tool was used. The learning rates were 0.001, and the pertaining and fine-tuning process was 0.1. Using the Contagio-CTU-UNB dataset, the classification tasks included 6 class and 8 class with the ROC curve value 0.99. Moreover, the study achieved a high rate of accuracy (i.e., 99.59%) in the binary classification. With the use of the deep belief network and probabilistic neural network, Zhao et al. [27] proposed an IDS framework. In their study, they used the KDD Cup'99 dataset for monitoring the efficiency of the intrusion detection model. The dataset was divided into 10% training and 10% testing dataset. The results demonstrated that the adopted method outperformed the other three models: (i) the traditional probabilistic neural network, (ii) principal component analysis with traditional probabilistic neural network, and (iii) optimized deep belief network with probabilistic neural network. Zhang et al. [28] attempted to design a self-adaptive model to modify the structure of the network enabling it to face different types of attacks. Thus, they presented an intrusion detection model based on both improved Genetic Algorithm (GA) and Deep Belief Network (DBN). DBN module is mainly divided into two steps in the training phase: (i) each RBM is trained separately, and (ii) the last layer of the DBN is set as the BP neural network. Using the NSL-KDD dataset, the performance of the proposed model showed a high detection rate of 99%. The main advantage of the intrusion detection system is recognizing malicious cyberattacks on a network. Besides that, the intrusion detection system can help in monitoring and evaluating the activities in a network or computer system [29, 30]. The area of cybersecurity has gained much attention from many researchers where they focused on developing systems that are able to detect security risks and prevent attacks. One of the well-known cybersecurity systems is the signature-based network intrusion detection system [31] which works by looking for specific patterns, for example, byte sequences in network traffic. This system has gained commercial success with widespread of applications. Another system which is regarded as superior to signature based is the anomaly-based system. This system has the ability to detect unknown attacks [32, 33]; it is based on machine learning which creates a model of trustworthy activity and compares new behavior against this model [34–36]. A shortcoming of this approach is that it may raise a false-positive alarm for previously unknown legitimate activity and classifying it as a malicious [32]. Therefore, developing intrusion systems with the ability to minimize the false-positive rates must be of primary concern. Hence, such issues can be solved by considering detection approaches based on machine learning. Machine learning is regarded as a discipline within artificial intelligence; other disciplines within artificial intelligence are computational statistics, data mining, and data science. Machine learning is based on the idea that computers can learn from data [36, 37]. It is closely related to mathematical theories, methods, statistical analysis, optimization, and many application areas in the field.

RETRACTED

Therefore, machine learning plays a primary role in the area of cybersecurity where building an intelligent security model for predictions is based on understanding the raw security data. It is known that the association analysis is considered in machine learning techniques for building rule-based intelligent systems [38–40]. However, in the current study, the main focus is on the learning techniques of classification [35, 41], which leverages a given training dataset for the sake of building a predictive system. For example, building a data-driven predictive model requires many techniques like naive Bayes classifier, support vector machines, k-nearest neighbors, logistic sigmoid function, and rule-based classification [35, 36]. Plenty of studies focused on detecting intrusions or cyberattacks and have used the abovementioned machine learning classification techniques. Li et al. [42] employed the hyperplane-based support vector machine classifier to classify identified attack categories, for example, DoS, Probe or Scan, U2R, R2L, and normal traffic leveraging the highly popular KDD'99 Cup dataset. Amiri et al. created faster systems through using a least-squared support vector machine classifier. This classifier helped in training the designed model with the use of large datasets [43].

Over the past five to ten years, nearly every company and organization has undergone a digital transformation through the adoption of cloud, mobile technologies, and the internet. These technologies have opened up new organizational capabilities. However, they created new complexities and vulnerabilities that, once cybercriminals learn about them, can quickly be exploited. A new wave of creative, sophisticated, and multichannel attacks floods companies with thousands of alerts, and hundreds of thousands of potential malicious files are analyzed every day. Currently, artificial intelligence based on the machine learning and deep learning algorithms for data-processing capabilities provides the most effective value to the areas of cyber defenses through uncovering patterns, shapes, and outliers that indicate potential incidents, even if these solutions do not align with known attack patterns. The current research contributes to the area of cybersecurity by developing a system based on the deep learning algorithm (LSTM-RNN) to detect an anomaly, thus making the system able to detect unknown attacks. The proposed system was tested and evaluated by using four standard network datasets and two types of attacks have been considered in developing the system, namely Denial-of-Service attack (DoS) and Distribute Denial-of-Dervice (DDoS).

## 2. Materials and Methods

Figure 1 displays the framework of the proposed system for detecting anomaly based on cybersecurity.

### 2.1. Datasets

In this experiment, the four standard datasets were conducted to test the proposed system for cybersecurity. The detailed description of these data is presented in the next subsubsections.

RETRACTED

#### 2.1.1. KDD Cup'99 Dataset

The KDD (Data Mining and Knowledge Discovery) cup dataset was developed for the intrusion detection system; it was represented in the 3rd international knowledge discovery and data mining and machine learning tools. These datasets were collected from Local-Area Network (LAN) by Lincoln Lab, which contains a record of around five million connection networks. It contains four major types of attacks: Denial of Service (DOS), Probe, User to Root (U2R) and Remote to Local (U2R) attacks, and 41 features. In this study, a deep learning algorithm was developed to detect the DoS attack. The dataset is available in the following link http://kdd.ics.uci.edu/databases/kddcup99/kddcup99.html.

#### 2.1.2. NSL-KDD Dataset

The NSL-KDD is an updated dataset of KDD Cup'99, developed by McHugh. It contains four major types of attacks: Denial of Service (DoS), Probe, User to Root (U2R) and Remote to Local (U2R), and 41 features. The dataset is available on this website: https://www.unb.ca/cic/datasets/index.html.

#### 2.1.3. ISCX Dataset

The ISCX2012 was gathered from the University of New Brunswick in 2012. This dataset consists of two profiles: the Alpha-profile, which carries out DDoS attacks, and the Beta-profile, which is the benign network traffic generator. The dataset has been collected from network traffic which contains different protocols like HTTP, SMTP, SSH, IMAP, POP3, and FTP. The dataset is available on this website: https://www.impactcybertrust.org/dataset_view?idDataset=916.

#### 2.1.4. CIC-IDS2017 Dataset

This dataset was collected from the Canadian Institute for cybersecurity. It contains benign networks generator and attacks, which looks like the true real-world data (PCAPs). The dataset was gathered in period starting at 9 a.m., Monday, July 3, 2017, and ended at 5 p.m. on Friday, July 7, 2017, for a total of 5 days. The normal network traffic collected on Monday. The network traffic included different types of protocols such as Brute Force FTP, Brute Force SSH, DoS, Heartbleed, Web Attack, Infiltration, Botnet, and DDoS. In this study, the Friday network traffic is considered for developing the deep learning system. It contains only DDoS attack and normal traffic. The dataset is available on https://www.unb.ca/cic/datasets/ids-2017.html.

### 2.2. Preprocessing

In this section, a detailed description of preprocessing techniques is presented. This is very important and significant in network traffic analysis, because the network traffic patterns have various types of format and dimensionality. Preprocessing is the main stage in data analysis; it is employed to manage real-world datasets into an intelligible format. Undoubtedly, most of the real-world datasets have been imperfect, noisy, and very difficult for determining the behavior of this data [44]. Preprocessing plays a vital role in analyzing patterns from network data for achieving accurate results. The information gain method was suggested to handle the important features from network datasets for detecting the malicious attacks.

RETRACTED

#### 2.2.1. Information Gain (IG)

Information gain, which is calculated based on information entropy, represents the degree of uncertainty of information elimination, and feature selection can be performed by sorting variables by the magnitude of information gain. The amount of information has a monotonically decreasing relationship with probability. The smaller the probability, the greater the amount of information. Information gain, that is, the reduced part of the prior entropy to the posterior entropy, reflects the degree of information elimination uncertainty [45]. The information gain method is one of the ranking feature selection methods which is used to score the variable by using a threshold method for removing variable below the value of the threshold.

(1) $$\begin{array}{c} H\left(Y\right)=-\underset{y\in Y}{\sum }P\left(y\right)\;\log_{2}\;\left(p\left(y\right)\right), \end{array}$$

where *H*(*Y*) is an entropy for cybersecurity datasets (*y*) which quantifies the uncertainty involved in the predictive value of a random variable.

(2) $$\begin{array}{c} H\left(Y/X\right)=-\underset{x\in X}{\sum }P\left(x\right)\underset{y\in Y}{\sum }P\left(\frac{y}{x}\right)\;\log_{2}\;\left(p\left(\frac{y}{x}\right)\right), \end{array}$$

where *H*(*Y*/*X*) is a condition entropy of the *x*, *p* and GI is information gain:

(3) $$\begin{array}{c} \text{GI}=H\left(Y\right)-H\left(\text{Y}/\text{X}\right) \end{array}$$

### 2.3. Machine Learning Algorithms

The traditional machine learning, namely Support Vector Machine (SVM) and K-Nearest Neighbor (K-NN), was presented to detect anomalies used in cybersecurity. The detailed description of classification algorithms is as follows:

#### 2.3.1. Support Vector Machine (SVM) Algorithm

Support Vector Machines (SVM) is a binary classification model. Its basic model is a linear classifier with the largest interval defined in the feature space. The largest interval makes it different from the perceptron. SVM also includes kernel techniques, which makes it an essential nonlinear classifier that is also equivalent to the problem of minimizing the regularized hinge loss function. The learning algorithm of SVM is the optimal algorithm for solving convex quadratic programming. The basic idea of SVM learning is to solve the separation hyperplane that can correctly divide the training dataset and have the largest geometric interval. For a linearly separable dataset, there are infinitely many such hyperplanes but the separating hyperplane with the largest geometric interval is the only one.

(4) $$\begin{array}{c} K\left(X,X^{\prime }\right)=\exp\left(-\frac{{\left\|X-X^{\prime }\right\|}^{2}}{2\sigma^{2}}\right), \end{array}$$

where the *X*, *X*′ are training data of the dataset and represent the features vectors of the input dataset and the ‖*X* − *X*′‖^2^ is the squared Euclidean distance between the two features input. The *σ* is a free parameter. Its decision boundary is the maximum margin for solving learning samples. SVM is one of the most robust and accurate methods among all well-known data mining algorithms. It belongs to a two-class classification algorithm and can support linear and nonlinear classification. In this research work, the Radial Basis Function (RBF) was applied to detect the malicious attacks.

RETRACTED

#### 2.3.2. K-Nearest Neighbor (K-NN) Algorithm

The KNN algorithm is classified by measuring the distance between different feature values. *K* is usually an integer not greater than 20. In the KNN algorithm, the selected neighbors are all objects that have been correctly classified. This method only determines the category of the sample to be classified based on the category of the nearest one or several samples in the decision-making of classification.

The K-nearest neighbor algorithm is used to find the *K* values that are close to values in the training dataset, and most of these K values belong to a certain class; then, the input instance is classified into this category.

(5) $$\begin{array}{c} D_{i}=\sqrt{\left(x_{1}-x_{2}\right)+{\left(y_{1}-y_{2}\right)}^{2}}. \end{array}$$

The *K* value is used to find the closet points in the feature vectors; the value should be a unique value.

#### 2.3.3. Long-Short Term Memory Recurrent Neural Network (LSTM-RNN)

Recurrent Neural Network (RNN) is one type of deep learning technique. The RNN model has a directional control loop which enables the previous states to be stored, recalled, and added to the current output [1, 2]. RNN has the gradient vanishing problem, so in order to sort out this problem, Long Short Memory (LSTM) is presented [46–48].  Figure 2 shows the structure of LSTM model for classifying the cyberattacks.

The hidden layer is referred to as *h*_*t*_, input as *x*_*t*_, and output as *y*_*t*_. In addition, the RNN has internal loops which perform a series of instructions for expressing the output as being a function of a past hidden layer besides being a function of a new input. In this way, the network continues growing. The RNN enables tackling the issue of exploding and vanishing, thus preserving information. The process of the cell state is supported by the RNN, which helps in the transmission of the input data into a certain network element, and then, they are integrated with subsequent element. RNN is different from the normal neural network where it can be visualized as multiple copies of a neural network; each passes information to the next one. The state of the cell is like a conveyer belt carrying the whole architecture of the network through the entire chain. The cells have gates, which have the function of regulating the information carried throughout the conveyer belt. These gates are composed of sigmoid type activation where the output gate value and *y*_*t*_ are subject of multiplication. The sigmoid function has the values of 0 and 1, where the 0 value represents the transition information and 1 value represents the whole information [49].

(6) $$\begin{array}{c} h_{t}=\text{sigm }\left(W_{xt}+{Uh}_{t-1}+b^{\left(h\right)}\right), \end{array}$$

(7) $$\begin{array}{c} O_{t}=\text{sigm }\left({Vh}_{t}+b^{\left(o\right)}\right), \end{array}$$

where *h*_*t*_ refers to the hidden layer that corresponds to the output *x*_*t*_, *h*_*t*_¯1 refers to the hidden state of recurrent neural network, *x*_*t*_ refers to the input data, and *O*_*t*_ refers to the output value. The weight vector of neural network is represented by *W*, *U*, and *V*. The *b* refers to the bias vector in a neural network. The structure of the long-short term memory cell is shown in Figure 3. The forget gate is represented as (*f*_*t*_), input gate (*i*_*t*_), input modulation gate (*m*_*t*_), output gate (*O*_*t*_), memory cell (*C*_*t*_), and hidden state (*h*_*t*_). The gates are computed:

(8) $$\begin{array}{c} f_{t}=\text{sigm }\left(W^{\left(f\right)}+X_{t}+U^{\left(f\right)}\;h_{t-1}+b^{\left(f\right)}\right), \end{array}$$

(9) $$\begin{array}{c} i_{t}=\text{sigm }\left(W^{\left(i\right)}+X_{t}+U^{\left(i\right)}\;h_{t-1}+b^{\left(i\right)}\right), \end{array}$$

(10) $$\begin{array}{c} m_{t}=\tanh\;\left(W^{\left(m\right)}+X_{t}+U^{\left(m\right)}\;h_{t-1}+b^{\left(m\right)}\right), \end{array}$$

(11) $$\begin{array}{c} o_{t}=\text{sigm }\left(W^{\left(o\right)}+X_{t}+U^{\left(o\right)}\;h_{t-1}+b^{\left(o\right)}\right), \end{array}$$

where *x*_*t*_ is a training input data, *W* and *U* are parameters used to adjust the weight matrices, and *h*_*t*−1_ is the previous hidden layer in the long-short term memory network. In order to transfer the data from input into output, the logistic sigmoid function is used. The hyperbolic tangent function is based on the tanh function, and the *b* is the bias vector of training data. We computed memory cell (*c*_*t*_) and hidden state (*h*_*t*_) by these equation:

(12) $$\begin{array}{c} c_{t}=i_{t}.m_{t}+f_{t}.c_{t-1}, \end{array}$$

(13) $$\begin{array}{c} h_{t}=o_{t}.\text{tahn }\left(c_{t}\right). \end{array}$$

In this research, the following specific structure of LSTM model was utilized to detect the cybersecurity attacks. Figure 3 shows LSTM model for cyberattack detection.

(14) $$\begin{array}{c} f\;\left(x\right)=\max\left(0,x\right). \end{array}$$

Sigmoid activation function is used to perform classification of the intrusion classes. The significant parameter values of LSTM model is presented in Table 1. The formula of sigmoid function is expressed as follows:

(15) $$\begin{array}{c} \sigma =\frac{\;1}{1-e^{2x}}. \end{array}$$

RETRACTED

## 3. Experiment Environment Setup

In order to develop a robust cybersecurity system for detecting the cyberattacks, we should provide answers for the following set of questions; this will grant developing a successful system.

1. Do the selected features score the highest ranking by using information methods?
2. Can these features help in reducing the negligible features that obstructed getting accurate results by the proposed system?
3. Do the advanced learning algorithms like deep learning have the ability to make the system more secure?
4. Why should we compare the results of the basic machine learning and the deep learning used in detecting cyberattacks?

The answers of the above questions begin by using four standard network datasets to test the proposed system. The proposed system focused on detecting the DoS and DDOS attacks from these datasets. For the selection purity of network features, the information gain method was applied. These important features can help to obtain the highest classification accuracy. The implementation of this research has been done by using Python 3.7 with tensor flow 1.14 library and Matlab 2018 programming. The experiments were conducted on the system with I5 Processor and 4 GB RAM to process all tasks of the system. The evaluation metrics were used to evaluate the proposed system.

### 3.1. Significant and Ranking Features Using Information Gain Method

To answer questions one and two, the feature selection method was used to handle the dimensionality reduction and select the subset features from the network dataset. The information gain method was applied for enhancing the accuracy of the classifying algorithms with less cost and time saving. 10 features were selected which scored the highest rank from KDD Cup'99, NSL-KDD, and CID-ID2017 datasets.  Figure 4 displays the significant selection features and their ranking obtained from information gain method for three datasets (KDD Cup'99, NSL-KDD, and CID-ID2017), whereas the ISCX dataset has 11 features. These features were considered to examine the proposed system for detecting cyberattacks.

RETRACTED

The information gain method was applied to select the significant features for improving the classification process. The information gain method depends on the ranking of the features that have lower entropy. In this research, four network datasets were considered to evaluate the proposed system, and two types of attacks were employed to test the efficiency of this system; these attacks are DoS and DDOS.  Table 2 shows the important features of KDD Cup'99 dataset. The KDD cup'99 dataset has 41 features in general, the highest ranking features obtained by information gain method were selected. The significant features of NSL-KDD dataset obtained by using information gain method are presented in Table 3. 10 important features were selected which have the highest ranking among the 41 features compared with another dataset features. The CIC-ID2017 dataset contains 78 features, we have selected the 10 important features using information gain method. The 10 significant features are shown in Table 4.  Figure 5 displays the ranking of KDD Cup'99, NSL-KDD, and CIC-ID2017 features of ICI-ID2017 dataset that were obtained by using information gain method.

### 3.2. Evaluation Metrics

In order to evaluate and measure the effectiveness of the proposed system to detect cyberattacks, the evaluation metrics like accuracy, sensitivity, specificity, precision, recall, and F1 score were employed. The equations are defined as follows:

(16) $$\begin{array}{c} \text{Accuracy}=\frac{\text{TP}+\text{TN}}{\text{FP}+\text{FN}+\text{TP}+\text{TN}}, \end{array}$$

(17) $$\begin{array}{c} \text{Specificity}=\frac{\text{TN}}{\text{TN}+\text{FP}}\times 100\%\text{Specifity}=\frac{\text{TN}}{\text{TN}+\text{FP}}\times 100\%, \end{array}$$

(18) $$\begin{array}{c} \text{Sensitivity}=\frac{\text{TP}}{\text{TP}+\text{FN}}\times 100\%\text{Sensivity}=\frac{\text{TP}}{\text{TP}+\text{FN}}\times 100\%, \end{array}$$

(19) $$\begin{array}{c} \text{Precision}=\frac{\text{TP}}{\text{TP}+\text{FP}}\times 100\%\text{Sensivity}=\frac{\text{TP}}{\text{TP}+\text{FN}}\times 100\%, \end{array}$$

(20) $$\begin{array}{c} \text{Recall}=\frac{\text{TP}}{\text{TP}+\text{FN}}\times 100\%, \end{array}$$

(21) $$\begin{array}{c} \text{F}1\text{ score}=2*\frac{\text{precision}*\text{Recall}}{\text{precision}*\text{Recall}}\;\times 100\%, \end{array}$$

where TP is true positive, FP is false positive, TN is true negative, and FN is false negative.

RETRACTED

### 3.3. Splitting of Datasets

The following table provides a description of the types of datasets used in these experiments.  Table 5 shows the splitting of the datasets.

## 4. Experimental Results

In this section, classification results of machine learning and deep learning based on the LSTM-RNN algorithm are presented. The empirical results of the system were examined by using the evaluative metrics: accuracy, sensitivity, specificity, precision, recall, and F1 score. The system was developed to detect the DoS and DDoS attacks. The classification algorithms were processed the significant features that have obtained from information gain method. The detailed description of the empirical results of the proposed system for detecting cyberattacks is presented in the following subsection.

### 4.1. Results of Machine Learning Algorithms

In this section, the results of machine learning, namely SVM and KNN algorithms, for detecting DoS and DDoS attacks are presented. The datasets were divided into 70% training and 30% testing. Tables 6 and 7 show the confusion matrix of SVM and KNN algorithms of four standard datasets. It is noted that the SVM algorithm results are better compared with the KNN algorithm.

The empirical results obtained from the machine learning approaches are calculated by making a confusion matrix. The confusion matrix reported the results of false positives, false negatives, true positives, and true negatives. Based on these numbers, the evaluation metrics namely accuracy, sensitivity, specificity, precision, recall, and F1 score are computed to test the proposed system.  Table 8 shows the empirical results of SVM algorithm to detect the DOS and DDOS attacks from network traffic. The prediction results of KNN algorithm is presented in Table 9. It is noted that both SVM and KNN algorithms have shown satisfactory results; nevertheless, the performance of the KNN algorithm is better with CIC-ID2017 dataset, whereas the SVM algorithm is better with KDD Cup'99 and NSL-KDD datasets. Finally, the SVM algorithm demonstrates slightly better performance over most datasets.

Figures 6 and 7 show the performance of the machine learning algorithms, namely SVM and KNN for detecting cyberattacks. It is observed that the machine learning algorithms are able to detect the normal and DoS and DDoS attacks from patterns in the network dataset according to the obtained results from unseen testing data.

### 4.2. Results of LSTM-RNN Algorithm

To answer the third question, the prediction results of deep learning based on the LSTM-RNN algorithm to detect the DoS, DDoS attacks and normal from standard network datasets are demonstrated. Experimental results were carried out on four different standard datasets.  Table 10 summarizes the confusion matrix of the LSTM-RNN algorithm.

RETRACTED

The confusion matrix reported the number of false positives, false negatives, true positives, and true negatives. For analyzing the classifications of the LSTM-RNN algorithm, we used dissimilar evaluation parameters along with their formulas as cited above. These are accuracy, sensitivity, specificity, precision, recall, and F1 score. While calculating these parameters, it is noticed that the proposed model provides better performance in all network datasets.  Table 11 shows the empirical results obtained from the LSTM-RNN algorithm.

Figure 8 shows the performance of LSTM-RNN model to classify the cyber-attack by using four standard network datasets. The graphical representation shows the validation result of the LSTM-RNN model and the number of epochs considered to run the system. Overall, the LSTM-RNN model achieved optimal results compared with traditional machine learning algorithms.

### 4.3. Results Discussion

To answer the fourth question, a comparative presentation of the prediction results of the traditional machine learning and deep learning based on LSTM-RNN algorithms is given in order to approve the effectiveness of the proposed system for detecting the cyberattacks. We use the same training and testing set of data for all the algorithms.

The result outcome from the machine learning, namely SVM and KNN and deep learning, based on the LSTM-RNN algorithms for detection cyber-attack is approved by using evaluation metrics. The empirical results were calculated using the confusion matrix obtained from the proposed model. We calculate the validation results only for finding the capability of the proposed system to identify the DOS and DDoS attacks. In order to save the time of building the model and the accuracy, the preprocessing method is important for handling the datasets features. The information methods were applied to select the highest ranking features and these features are significant for detecting cyberattacks. These features were processed by using the machine learning and LSTM algorithms; it is noted that the LSTM-RNN model has achieved the highest accuracy over all the network datasets. The LSTM-RNN model gave significant results in terms of accuracy, sensitivity, specificity, precision, recall, and F1 score which ensures the model effectiveness while predicting anomalies or intrusions. In addition, Figure 9 shows the outcome results of the LSTM-RNN against the machine learning SVM and KNN algorithms in terms of accuracy values.

## 5. Conclusion

In this paper, we presented the machine learning and deep learning algorithms to detect anomalies in cybersecurity attacks. Taking into account the multidimensional nature of the network features due to the different formats of the network dataset, we find the preprocessing stage is very important to handle this multidimensionality. Furthermore, the information gain method was applied to select the highest ranking network features for building the system. For making the system more secure, we selected the important network features. These features were processed by classifying algorithms to detect the anomaly in the cybersecurity attacks. The machine learning algorithms like SVM and KNN algorithms and deep learning based on the LSTM-RNN model were implemented. The effectiveness of the proposed system was examined by conducting a number of experiments on cybersecurity datasets. The proposed system was tested by using evaluation metrics for unseen dataset. The experimental results showed the effectiveness of the proposed system to detect the intrusion attacks on cybersecurity. Overall, deep learning based on the LSTM-RNN algorithm achieved the highest accuracy. Comparison of outcome results of LSTM-RNN model with traditional machine learning approaches for analyzing the effectiveness of these approaches is also presented. In a future work, we will apply the propped system in Internet of Things (IoT) security services on cybersecurity attacks.

RETRACTED

## Figures and Tables

**Figure 1:** Framework for proposed methodology.

**Figure 2:** Structure of LSTM model.

**Figure 3:** LSTM model for cyberattack detection.

**Figure 4:** The significant features with ranking values from the datasets.

**Figure 5:** Performance of information gain method (a) KDD Cup'99, (b) NSL-KDD, and (c) CIC-IDS 2017 datasets.

**Figure 6:** Performance of SVM algorithm of testing results to classify cyberattacks.

**Figure 7:** Performance of KNN algorithm of testing results to classify anomaly based on cyberattacks.

**Figure 8:** Performance of LSTM-RNN model for testing data.

**Figure 9:** Comparison of the LSTM-RNN against machine learning algorithms in terms of accuracy metric.

**Table 1:** Parameter values of LSTM model used in the proposed system.

Parameter name	Values
LSTM units	32
Drop out	0.2
Dense feed forward layer (DFFL)	265
Dense output layer	2
Epochs	10
Batch size	205

**Table 2:** Top ranked features of KDD Cup'99 using information gain method.

Feature's number	Feature's name
f26	srv_serror_rate
f29	same_srv_rate
f36	dst_host_same_src_port_rate
F40	dst_host_rerror_rate
F35	dst_host_diff_srv_rate
F23	Count
F9	Urgent
F32	diff_srv_rate
F29	dst_host_srv_count
F21	host_login

**Table 3:** Top ranked features of NSL-KDD using information gain method.

Feature's number	Feature's name
F5	src_bytes
F3	Service
F32	dst_host_srv_count
F25	serror_rate
F37	dst_host_serror_rate
F39	dst_host_rerror_rate
F26	srv_serror_rate
F29	same_srv_rate
F23	Count
F24	srv_coun

RETRACTED

**Table 4:** Top ranked features of CIC-ID2017 using information gain method.

Feature's number	Feature's name
F15	Flow bytes/s
F16	Flow packets/s
F41	Packet length mean
F11	Bwd packet length max
F40	Max packet length
F13	Bwd packet length mean
F55	Avg Bwd segment size
F42	PSH flag count
F14	Bwd packet length Std
F53	Average packet size

**Table 5:** Distribution and splitting of the used datasets.

Dataset name	Total of samples	Training set (70%)	Testing set (30%)	Total of normal class	Total and type of attack class
KDD Cup'99	133193	93235	39958	1131107	2086 DDOS attack
NSL-KDD	29175	20422	8753	15601	13574 DOS attack
ISCX	24431	17101	7330	18426	6005 DOS attack
CIC-ID2017	19933	13953	5980	11833	8100

**Table 6:** Confusion matrix of SVM algorithm.

Datasets	True positive	False positive	True negative	False negative
KDD Cup'99	39331	9	615	3
NSL-KDD	4508	151	3941	153
ISCX	1773	5	5413	139
ICI-ID2017	2313	1265	2396	4

**Table 7:** Confusion matrix of KNN algorithm.

Datasets	True positive	False positive	True negative	False negative
KDD Cup'99	39222	124	500	112
NSL-KDD	3918	865	3754	216
ISCX	5553	1	1774	2
ICI-ID2017	2382	43	3515	40

**Table 8:** Testing results of SVM algorithm.

	Accuracy (%)	Sensitivity (%)	Specificity (%)	Precision (%)	Recall (%)	F1 score (%)	Time (second)
KDD Cup'99	99.97	99.98	99.51	99.99	99.98	99.98	85.22
NSL-KDD	96.53	96.76	96.26	96.72	96.72	96.76	286.67
ISCX	98.03	99.71	97.49	92.73	99.71	96.09	34.53
ICI-ID2017	78.77	64.64	99.83	99.98	64.64	78.47	78.18

**Table 9:** Testing results of KNN algorithm.

	Accuracy (%)	Sensitivity (%)	Specificity (%)	Precision (%)	Recall (%)	F1 score (%)	Time (second)
KDD Cup'99	99.40	99.71	81.69	99.68	81.69	99.70	255.42
NSL-KDD	87.65	81.27	94.77	94.55	81.27	87.41	168.09
ISCX	99.95	99.94	99.64	99.88	99.94	99.91	94.83
ICI-ID2017	98.61	98.79	98.35	98.79	98.83	98.57	53.67

**Table 10:** Confusion matrix of LSTM-RNN algorithm.

	True positive	False positive	True negative	False negative
KDD Cup'99	39284	74	600	0
NSL-KDD	4288	366	3901	198
ISCX	5552	6	1769	3
ICI-ID2017	3576	6	2340	58

**Table 11:** Testing results of LSTM-RNN algorithm.

	Accuracy (%)	Sensitivity (%)	Specificity (%)	Precision (%)	Recall (%)	F1 score (%)	Time (second)
KDD Cup'99	99.81	100	89.02	99.78	100	99.90	120.60
NSL-KDD	93.55	95.58	91.42	92.13	95.58	93.82	48.20
ISCX	99.87	99.94	99.66	99.89	99.94	99.91	40.25
CIC-ID2017	98.92	98.40	99.74	99.83	98.40	99.11	68.12

## Data Availability

The KDD (Data Mining and Knowledge Discovery) cup dataset was developed for the intrusion detection system; it was represented in the 3rd international knowledge discovery and data mining and machine learning tools. These datasets were collected from Local-Area Network (LAN) by Lincoln Lab, which contains a record of around five million connection networks. It contains four major types of attacks: Denial of Service (DOS), Probe, User to Root (U2R) and Remote to Local (U2R) attacks, and 41 features. In this study, a deep learning algorithm was developed to detect the DoS attack. The dataset is available in the following link http://kdd.ics.uci.edu/databases/kddcup99/kddcup99.html. In “NSL-KDD Dataset” subsubsection, the NSL-KDD is an updated dataset of KDD Cup'99, developed by McHugh. It contains four major types of attacks: Denial of Service (DoS), Probe, User to Root (U2R) and Remote to Local (U2R), and 41 features. The dataset is available on this website: https://www.unb.ca/cic/datasets/index.html. In “ISCX Dataset” subsubsection, the ISCX2012 was gathered from University of New Brunswick in 2012. This dataset consists of two profiles: the Alpha-profile, which carries out DDoS attacks, and the Beta-profile, which is the benign network traffic generator. The dataset has been collected from network traffic which contains different protocols like HTTP, SMTP, SSH, IMAP, POP3, and FTP. The dataset is available on this website: https://www.impactcybertrust.org/dataset_view?idDataset=916. In “CIC-IDS2017 Dataset” subsubsection, this dataset was collected from the Canadian Institute for cybersecurity. It contains benign networks generator and attacks, which looks like the true real-world data (PCAPs). The dataset was gathered in period starting at 9 a.m., Monday, July 3, 2017, and ended at 5 p.m. on Friday, July 7, 2017, for a total of 5 days. The normal network traffic collected on Monday. The network traffic included different types of protocols such as Brute Force FTP, Brute Force SSH, DoS, Heartbleed, Web Attack, Infiltration, Botnet, and DDoS. In this study, the Friday network traffic is considered for developing the deep learning system. It contains only DDoS attack and normal traffic. The dataset is available on https://www.unb.ca/cic/datasets/ids-2017.html.
